The article "MicroRNA-379 inhibits the proliferation, migration and invasion of human osteosarcoma cells by targetting EIF4G2" was retracted in 2021. Reasons: duplicated images; signs of a paper mill.

# MicroRNA-379 inhibits the proliferation, migration and invasion of human osteosarcoma cells by targetting EIF4G2

**DOI:** 10.1042/BSR20160542

**Published:** 2017-05-17

**Authors:** Xi Xie, Yu-Sheng Li, Wen-Feng Xiao, Zhen-Han Deng, Hong-Bo He, Qing Liu, Wei Luo

**Affiliations:** 1 Department of Orthopedics, Xiangya Hospital, Central South University, Changsha 410008, P.R. China; 2 Department of Day Surgery Center, Xiangya Hospital, Central South University, Changsha 410008, P.R. China

**Keywords:** EIF4G2, Invasion, MicroRNA-379, Migration, Osteosarcoma, Proliferation

## Abstract

Osteosarcoma (OS) is an aggressive malignant mesenchymal neoplasm amongst adolescents. The aim of the present study was to explore the various modes of action that *miR-379* has on the proliferation, migration, and invasion of human OS cells. *miR-379* achieves this by targetting eukaryotic initiation factor 4GII (EIF4G2). Human OS cell lines U2OS and MG-63 were selected and assigned into blank, *miR-379* mimics, *miR-379* mimic negative control (NC), *miR-379* inhibitors, *miR-379* inhibitor NC, EIF4G2 shRNA, control shRNA, and *miR-379* inhibitor + EIF4G2 shRNA group. The *miR-379* expression and *EIF4G2* mRNA expression were detected utilising quantitative real-time PCR (qRT-PCR) and the EIF4G2 protein expression using Western blotting. MTT assay, scratch test, Transwell assay, and flow cytometry were performed to determine the proliferation, migration, invasion, and cell cycle, respectively. In comparison with the *miR-379* mimic NC group, the *miR-379* mimics group had decreased EIF4G2 expression; the *miR-379* inhibitors group indicated an increased EIF4G2 expression. Compared with the control shRNA group, the EIF4G2 expression was lower in the EIF4G2 shRNA group and the *miR-379* expression was dropped in the *miR-379* inhibitor + EIF4G2 shRNA group. The proliferation, migration, and invasion abilities of OS cells were reduced in the *miR-379* mimics and EIF4G2 shRNA groups. The percentage of OS cells at the G_0_/G_1_ stage was increased, and the percentage at the S-stage was decreased in the *miR-379* mimics and EIF4G2 shRNA groups. *miR-379* may inhibit the proliferation, migration and invasion of OS cells through the down-regulation of EIF4G2.

## Introduction

Osteosarcoma (OS) is the most common primary malignancy and is derived from the primitive bone-forming mesenchymal cells in the long bones [1]. OS commonly occurs in adolescents between the ages of 10 and 20, while accounting for 8.9% of cancer deaths amongst children and adolescents in the United States alone. There appears to be no significant difference in gender, however, the incidence of OS varies with ethnicity [2]. Currently, the most common treatment available for OS is pre- and post-operational chemotherapy in association with surgical treatment [3]. Unfortunately, despite advancements in the diagnosis and treatment of OS, the overall survival rate amongst patients has dithered and remained relatively constant since the mid 1980s [4]. Universal common risk factors linked to OS development include ionising radiation, alkylating agents, Paget’s disease, hereditary retinoblastoma, the Li–Fraumeni familial cancer syndrome and other chromosomal abnormalities [2]. Recently, genetic aberrations have received increasing recognition as a key factor in the etiology of OS [2].

miRNAs (miRs) are a class of small non-coding (18–24 nts) RNAs [5]. miRs regulate gene expression by inducing mRNA degradation and/or repressing translation and therefore participate in a number of biological processes, such as development, cell proliferation, differentiation, and apoptosis [1,6]. *miR-664* promotes the proliferation of OS cells through the down-regulation of FOXO4 [7]. Down-regulated *miR-125a-5p* suppresses OS by targetting MMP-11 [8]. It has been shown that *miR-155-5p* and *miR-148a-3p* are species conserved deregulated miR in OS [9]. *miR-379* is located on chromosome 14q32.31 and belongs to the δ-like 1 homolog-deiodinase, iodothyronine 3 (DLK1-DIO3) clusters [10,11]. The DLK1-DIO3 miR clusters have been reported to play a critical role in regulating tumor growth and metastasis as well as driving tumor progression [12]. In addition, members of the clusters, *miR-379, miR-409-3p/5p*, and miR-154* have previously been extensively evaluated and have been shown to have a correlation to bone metastasis in prostate cancer [11,13]. A recent study highlighted that *miR-409-3p* may play a role in the inhibition of OS cell invasion and migration through targetting catenin-δ1 [14]. Limited studies have investigated the role of *miR-379* in OS and its underlying molecular mechanisms. Consequently, the hypothesis of the present study relates to emphasising the role of *miR-379* in OS. During the present study, an investigation into the effects of *miR-379* was made. The effects of *miR-379* on the proliferation, migration, and invasion of OS cells, through targetting eukaryotic initiation factor 4GII (EIF4G2) was explored in depth. This was done in addition to its under examined role in the development of OS.

## Materials and methods

### Cell recovery, culture, and grouping

The human OS cell lines U2OS and MG-63 were purchased from the Institute of Biochemistry and Cell Biology (Shanghai, China). The cell suspension and Dulbecco’s minimum essential medium (DMEM) were lightly mixed, followed by centrifugation for a 5-min period at 1000 rpm. After discarding the supernatant, the cells were resuspended in DMEM (5 ml) containing 10% FBS and transferred into a T25 culture flask. This was then placed in an incubator at 37°C with 5% CO_2_. According to the growth condition, the culture medium was replaced 2–3 days later. The cells were subcultured after reaching 80–90% confluence. After discarding the medium, the cells were washed twice with PBS, digested for 2–5 min with 0.25% trypsin, suspended in DMEM (5 ml) containing 10% FBS and passaged at a ratio of 1:2–3. The U2OS and MG-63 cells were divided into the blank group (transfected with blank plasmids), the *miR-379* mimics group (transfected with *miR-379* mimics), the *miR-379* mimic NC group (transfected with *miR-379* mimic negative control (NC)), the *miR-379* inhibitors group (transfected with *miR-379* inhibitors), the *miR-379* inhibitor NC group (transfected with *miR-379* inhibitors NC), the EIF4G2 shRNA group (transfected with EIF4G2 shRNA), the control shRNA group (transfected with control shRNA) and the *miR-379* inhibitor + EIF4G2 shRNA group (transfected with *miR-379* inhibitors and EIF4G2 shRNA), of which the plasmid sequences were shown in Table 1.

**Table 1:** The sequences of plasmids

Plasmid	Sequence
*miR-379* mimics	5′-UGGUAGACUAUGGAACGUAGG-3′
*miR-379* mimics NC	5′-GUGGAUUUUCCUCUAUGAUUU-3′
*miR-379* inhibitors	5′-ACAACAAAAUCACUAGUCUUCCA-3′
*miR-379* inhibitors NC	5′-ACAACAAAAUCACAAGUCUUCCA-3′
Control shRNA	5′- GCTCTGGAGCAGTTCCGATATC-3′
EIF4G2 shRNA	5′- CACTGAGGCTGAGCGAAAT-3′

### Cell transfection

The U2OS and MG-63 cells in the logarithmic growth phase were cultured in a 24-well plate with 2 × 6^5^ cells per well overnight. When the density of cells reached 70–90%, 0.8 g plasmids were added into 50 μl Opti-MEM and 2 μl Lipofectamine 2000 was added into another 50 μl Opti-MEM. After 5 min at room temperature, the two compounds were mixed and incubated for 20 min. Then the mixture was added into a 24-well plate and the medium was replaced after transfection for 4–6 h. The experiment in each group was repeated three times.

### Quantitative real-time polymerase chain reaction

After a 24-h period of transfection, the RNA of the transfected U2OS and MG-63 cells was extracted using TRIzol. UV spectrophotometer was used to determine the purity and concentration of the extracted RNA, and agarose gel electrophoresis was used to detect the completeness of the extracted RNA. A Primescript™ RT reagent kit (TaKaRa Biotechnology Ltd., Dalian, China) was used for reverse transcription and a SYBR® Premix Ex Taq™ quantitative real-time PCR (qRT-PCR) Kit (TaKaRa Biotechnology Ltd., Dalian, China) was used for PCR amplification. The sequences of primers are illustrated in Table 2. The Opticon Monitor 3 software (Bio–Rad Laboratories, Inc. CA, U.S.A.) was used to analyze the results of the PCR. The lowest point of the parallel rising logarithmic amplification curve was selected manually, as the threshold value and the cycle threshold (*C*_t_) for each reaction tube was obtained. Data were analyzed using the 2^−ΔΔ*C*^_t_ methods, referring to the odds ratio (OR) of the target gene expression, between the experimental group and the control group. The formula was as follows: ΔΔ*C*_t_ = (*C*_t__ target gene_ – *C*_t__the reference gene_) _ experimental group_ – (*C*_t__target gene_ – *C*_t__reference gene_) _ control group_. The experiment in each group was repeated three times. The comparison amongst the groups was analyzed by *t* test.

**Table 2:** Primer sequences for qRT-PCR

Gene	Sequence
*EIF4G2*	F: 5′-CCCTTCAAGATGCACCTCAT-3′
	R: 5′-GTGGTCCACAGCATTTCCTT-3′
*β-actin*	F: 5′-AGGGGCCGGACTCGTCATACT-3′
	R: 5′-GGCGGCACCACCATGTACCCT-3′
*miR-379*	F: 5′-GTGGTAGACTATGGAACGTAGG-3′
	R: 5′-TACGTTCCATAGTCTACCA-3′
*U6*	F: 5′-CTCGCTTCGGCAGCACA-3′
	R: 5′-AACGCTTCACGAATTTGCGT-3′

*n*=3; F, forward; R, reverse.

### Western blotting

After 24 h of transfection, cells were scraped from the ice, centrifuged at 3000 rpm at 4°C, added with RIPA (1:5) for proteolytic cleavage and placed in a refrigerator at 4°C for 1 h. Followed by centrifugation at 10000×***g*** for 30 min in a refrigerated centrifuge, the supernatant was transferred to a new EP tube and BCA kit (Univ-bio, Shanghai, China) was used to detect the concentration of proteins. With SDS/PAGE at 70 V for 120 min, the total protein (50 μg) was transferred to PVDF membrane. After blocking by using 5% skimmed milk at room temperature for 1.5 h, the membranes were incubated with the primary antibodies including anti-rabbit EIF4G2 antibody (1:1000, ab697302, Abcam Inc., MA, U.S.A.) and GAPDH antibody (1:2000, ab697302, Abcam Inc., MA, U.S.A.) This was conducted over a 2-h period and at a temperature of 4°C overnight. Membranes were washed with TBST (pH =7.4) three times and incubated with goat anti-rabbit IgG (1:2000) labeled with horseradish peroxidase at room temperature for 1 h. The images were scanned after development using ECL reagent. The gray values were analyzed by Image software. The relative expression of proteins resulted in the gray value of the target protein/the gray value of reference protein. The experiment in each group was repeated three times. The comparison amongst the groups was statically analyzed using a *t* test.

### Dual luciferase reporter gene assay

The biological prediction website microRNA.org was used to analyze target genes of *miR-379* and also to verify whether EIF4G2 was a direct target gene of *miR-379*. After cloning and amplifying the full length of EIF4G2 in 3′-UTR region, the PCR products were cloned into multiple cloning sites of pmirGLO luciferase (Promega Corp., Madison, WI, U.S.A.), which was named pEIF4G2-Wt. Site-specific mutagenesis was performed to alter the binding site of *miR-379*, which was predicted by bioinformatics, followed by construction of the pEIF4G2-Wt vector. The number of cells and transfection efficiency were normalized using pRL-TK (TaKaRa Biotechnology Ltd., Dalian, China) as an internal reference, which expressed *Renilla* luciferase. *miR-379* mimics and *miR-379* mimic NC were respectively cotransfected with the luciferase reporter vector into U2OS and MG-63 cells, followed by dual luciferase activity detection according to the instructions given by Promega. The experiment in each group was repeated three times. The comparison among the groups was analyzed by *t* test.

### MTT assay

Cell viability curves were drawn using MTT assay to measure the proliferation of the transfected U2OS and MG-63 cells. After 48 h of transfection, cells in each group were counted and then inoculated into four 96-well plates at a density of 2 × 10^2^ cells per 200 μl with eight repeated wells. Four time points were chosen: 0, 24, 48, and 72 h, and further experiments were performed at each time point. The MTT solution (20 μl) was added to each well for 4 h of incubation at 37°C, the incubation was then terminated and the culture supernatant was discarded. DMSO (150 μl) (Sigma, Englewood Cliffs, NJ, U.S.A.) was added to each well, and the plates were gently shaken for 10 min in an enzyme-linked immunosorbent detector. The absorbance (OD) values of each well were determined at a wavelength of 490 nm at each time point. Cell viability curves were generated with time as the *x*-axis and the OD value as the *y*-axis. The experiment in each group was repeated three times. The comparison amongst the groups was analyzed by *t* test.

### Scratch test

The cells were digested and the cell concentration was adjusted to 5 × 10^5^/ml. The cell suspension (100 μl) was added to a 24-well culture plate for conventional incubation until the formation of a cell monolayer. The scratch test was then performed. After washing once, the culture medium was replaced by RPMI 1640 BSA and 1% FBS, followed by measuring the distance of the scratch area under a microscope. After incubation for 24 h, the cells were cultured for another 24 h in RPMI 1640 culture medium with 10% FBS, followed by measuring the relative distance that the cells migrated to the injured area. Cell migration distance = scratch distance at the beginning of the experiment – scratch distance at the end of the experiment. The experiment in each group was repeated three times. The comparison amongst the groups was analyzed by *t* test.

### Transwell assay

Following transfection for 24 h, the cells were starved for 12 h and then digested in a serum-free medium, followed by washing twice with PBS and suspension in the serum-free medium Opti-MEMI (Invitrogen Inc., Carlsbad, CA, U.S.A.) with 10 g/l BSA. The cell density was adjusted to 3 × 10^4^ cells/ml. The experiment was performed in 24-well 8 μm Transwell plates (Corning-Costar, Corning, NY, U.S.A.) (three chambers per group; 100 μl cell suspension per chamber). The lower chamber, containing 600 μl 10% RPMI 1640 medium, was incubated in 5% CO_2_ at 37°C. Twenty-four hours later later, the cells were fixed with 4% paraformaldehyde for 30 min and 0.2% Triton X-100 (Sigma Company, St. Louis, MO, U.S.A.) solution was added to the chambers for 15 min, followed by 0.05% Gentian Violet staining for 5 min. Before the assay, 50 μl Matrigel (Sigma Company, St. Louis, MO, U.S.A.) was added to the chambers, and 48 h later, the chambers were fixed and stained using the method described above. The number of stained cells was counted under an inverted microscope. Five fields were randomly selected and the number of cells was represented as the mean. The experiment in each group was repeated three times. The comparisons amongst the groups were analyzed using a *t* test.

### Flow cytometry

The cells were transfected and cultured for 24 h. The cells were then washed with PBS solution once, after the culture solution was discarded. The cells were then digested by 0.25% trypsin solution, and the digestion liquid was discarded after the cells were contracted and turned around, which was observed under a microscope, followed by the addition of culture solution containing serum to help stop the digestion. Methodically pipetting, the cells were gently detached from the wall and mixed into cell suspension, which was then centrifuged (1000 rpm) for 5 min with a supernatant sucking technique. The cells were washed with PBS solution twice, and then fixed for 30 min by adding pre-cooled 70% ethanol. The cells were centrifuged and collected, washed with phosphate buffer, stained by 1% Propidium Iodide (PI) containing RNA enzyme for 30 min and washed with PBS solution twice for the elimination of PI. The volume was adjusted to 1 ml using PBS solution. The cell cycle was detected using a BD-Aria FACS Calibur flow cytometry, with three samples in each group. Detection was repeated three times uniformly. The comparison amongst the groups was analyzed using *t* test.

### Statistical analysis

SPSS 21.0 software (SPSS Inc., Chicago, IL, U.S.A.) was used for statistical analysis. Counting data were represented as rates and/or percentages. Comparisons were performed using a chi-square test. Measurement data were represented as mean ± S.D., and comparisons between the two groups were performed using a *t* test. Comparisons in multiple groups were performed using one-way ANOVA (variance homogeneity was tested before analysis). Comparisons between the two means were verified using the least significant difference *t* (LSD-*t*) test. A two-tailed *P*-value less than 0.05 was considered statistically significant.

## Results

### *miR-379* down-regulated EIF4G2 expression in U2OS and MG-63 cell lines

The results collected from qRT-PCR as well as Western Blotting (Figure 1) indicated that in the U2OS and MG-63 cell lines, no significant differences were found in the expressions of *miR-379* and EIF4G2 amongst the *miR-379* mimic NC, *miR-379* inhibitor NC, control shRNA and blank groups (all *P*>0.05). In comparison with the *miR-379* mimic NC group, the *miR-379* mimics group showcased a considerably increased rate if *miR-379* expression and decreased EIF4G2 expression (both *P*<0.05), while the *miR-379* inhibitors group, had decreased *miR-379* expression and increased EIF4G2 expression in relation to the *miR-379* inhibitor NC group (both *P*<0.05).

**Figure 1:** *miR-379* inhibited EIF4G2 expression in U2OS and MG-63 cell lines. (**A**) *miR-379* inhibited EIF4G2 expression in U2OS cells; (**B**) *miR-379* inhibited EIF4G2 expression in MG-63 cells; (**C**) the protein expression of EIF4G2 in U2OS cells in each group; (**D**) values of the protein expression of EIF4G2 in U2OS cells in each group; (**E**) the protein expression of EIF4G2in MG-63 cells in each group; (**F**) values of the protein expression of EIF4G2 in MG-63 cells in each group; *n*=3; *, *P*<0.05 compared with the *miR-379* mimic NC group; #, *P*<0.05 compared with the *miR-379* inhibitor NC group; @, *P*<0.05 compared with the control shRNA group.

In comparison with the control shRNA group, the EIF4G2 expression was lower in the EIF4G2 shRNA group (*P*<0.05) There was no significant difference between *miR-379* expression (*P*>0.05) The *miR-379* expression was dropped in the *miR-379* inhibitor + EIF4G2 shRNA group (*P*<0.05) and there was no significant difference in EIF4G2 expression (*P*>0.05). The correlation analysis indicated that *miR-379* was negatively correlated with regard to EIF4G2.

### *miR-379* targetted EIF4G2

A biological prediction website (microRNA.org) showed that *miR-379* could target EIF4G2 (Figure 2A). To confirm that EIF4G2 was a direct target gene of *miR-379*, the luciferase reporter vectors pEIF4G2-Wt and pEIF4G2-Mut were constructed using the EIF4G2 3′-UTR. The dual luciferase reporter assay showed that in U2OS cells, the luciferase activity in the *miR-379* mimics + pEIF4G2-wt group decreased by approximately 42% compared with that in the *miR-379* mimic NC group (all *P*<0.05) (Figure 2B), while the luciferase activity in the pEIF4G2-mut cells showed no difference between the *miR-379* mimics group and the *miR-379* mimic NC group (both *P*>0.05). In MG-63 cells, the luciferase activity in the *miR-379* mimics + pEIF4G2-wt group decreased by approximately 54% compared with that in the *miR-379* mimic NC group (all *P*<0.05) (Figure 2B), while the luciferase activity in the pEIF4G2-mut cells showed no difference between the *miR-379* mimics group and the *miR-379* mimic NC group (both *P*>0.05). Therefore, EIF4G2 was a potential target gene of *miR-379*, and *miR-379* could target and negatively regulate EIF4G2.

**Figure 2:** Identification of the targetting relationship between *miR-379* and EIF4G2 by bioinformatics analysis and dual luciferase reporter gene assay. (**A**) *miR-379* was predicted to target EIF4G2 by bioinformatics software; (**B**) dual luciferase reporter analysis verified the targetting relationship between *miR-379* and EIF4G2; *n*=3; *, *P*<0.05 compared with the *miR-379* mimic NC group.

### *miR-379* decreased the proliferation of U2OS and MG-63 cells

Cell viability curves were drawn using the MTT method to determine the proliferation of the transfected U2OS and MG-63 cells. The OD values measured in the transfected cells were summarized in Figure 3A,B. The results showed that the U2OS and MG-63 cells transfected with *miR-379* mimics had a significantly slower growth rate than those transfected with *miR-379* mimic NC (all *P*<0.05). The growth rates of the cells in the blank, *miR-379* mimic NC, *miR-379* inhibitor NC, control shRNA and *miR-379* inhibitor + EIF4G2 shRNA groups were not significantly different (all *P*>0.05), while the growth rate of the cells was higher in the *miR-379* inhibitors group than that in the *miR-379* inhibitor NC group (all *P*<0.05). Compared with the control shRNA group, the growth rate of the cells was lower in the EIF4G2 shRNA group (all *P*<0.05).

**Figure 3:** The proliferation of U2OS and MG-63 cell lines detected by MTT assay. (**A**) The proliferation of U2OS cells in each group; (**B**) the proliferation of MG-63 cells in each group; *n*=3; #, *P*<0.05 compared with the *miR-379* inhibitor NC group; *, *P*<0.05 compared with the *miR-379* mimic NC group; @, *P*<0.05 compared with the control shRNA group.

### *miR-379* inhibited the migration of U2OS and MG-63 cells

Figure 4 showed the effects of *miR-379* on the migration of the U2OS and MG-63 cells. Using the scratch test, in the U2OS and MG-63 cells, the migration distances were (435.22 ± 22.83) and (412.72 ± 19.10) μm in the *miR-379* mimics group, (624.45 ± 15.41) and (620.03 ± 18.23) μm in the control shRNA group, (755.15 ± 18.49) and (738.72 ± 19.31) μm in the *miR-379* inhibitors group, (634.70 ± 19.22) and (601.71 ± 17.77) μm in the *miR-379* mimic NC group, (636.32 ± 14.12) and (611.30 ± 12.82) μm in the *miR-379* inhibitor NC group, (400.53 ± 20.65) and (390.76 ± 18.96) μm in the EIF4G2 shRNA group, (648.85 ± 14.27) and (638.76 ± 14.86) μm in the *miR-379* inhibitor + EIF4G2 shRNA group and (632.41 ± 14.41) and (629.76 ± 15.26) μm in the blank group. There was no significant difference in the migration distance in the U2OS and MG-63 cells amongst the blank, *miR-379* mimic NC, *miR-379* inhibitor NC, control shRNA and *miR-379* inhibitor + EIF4G2 shRNA groups (all *P*>0.05). Compared with the *miR-379* mimic NC group, the *miR-379* mimics group had a considerably reduced migration ability rate (*P*<0.05), while cell migration was significantly enhanced in the *miR-379* inhibitors group when compared with the *miR-379* inhibitor NC group (*P*<0.05). In relation to the control shRNA group, the migration ability of the cells was decreased in the EIF4G2 shRNA group (*P*<0.05).

**Figure 4:** The migration of U2OS and MG-63 cell lines detected by the scratch test. (**A**) The migration distance of the U2OS cells in each group; (**B**) observation of the migration ability of the U2OS cells under a light microscope; (**C**) the migration distance of the MG-63 cells in each group; (**D**) observation of the migration ability of the MG-63 cells under a light microscope; *n*=3; #, *P*<0.05 compared with the *miR-379* inhibitor NC group; *, *P*<0.05 compared with the *miR-379* mimic NC group; @, *P*<0.05 compared with the control shRNA group.

### *miR-379* reduced the invasion of U2OS and MG-63 cells

Figure 5A–H illustrates the effects of *miR-379* on the migration and invasion ability of the U2OS and MG-63 cells. There were no significant differences amongst the *miR-379* mimic NC, *miR-379* inhibitor NC, control shRNA and *miR-379* inhibitor + EIF4G2 shRNA and blank groups (all *P*>0.05). In comparison with the *miR-379* mimic NC group, the *miR-379* mimics group showed a significantly reduced migration and invasive ability (all *P*<0.05), while the *miR-379* inhibitors group showed significantly increased migration and invasion than the *miR-379* inhibitor NC group (all *P*<0.05). Compared with the control shRNA group, the migration and invasive ability of the cells were reduced in the EIF4G2 shRNA group (*P*<0.05).

**Figure 5:** The migration and invasion abilities of U2OS and MG-63 cell lines detected by the Transwell assay (**A**) The number of invasive U2OS cells in each group; (**B**) images of the invasion of U2OS cells under a light microscope; (**C**) the number of invasive MG-63 cells in each group; (**D**) images of the invasion of the MG-63 cells under a light microscope; (**E**) the number of migrating U2OS cells in each group; (**F**) images of the migration of U2OS cells under a light microscope; (**G**) the number of migrating MG-63 cells in each group; (**H**) images of the migration of the MG-63 cells under a light microscope; *n*=3; #, *P*<0.05 compared with the *miR-379* inhibitor NC group; *, *P*<0.05 compared with the *miR-379* mimic NC group; @, *P*<0.05 compared with the control shRNA group.

### Effect of *miR-379* on cell cycle of U2OS and MG-63 cells

Figure 6A,B showed the results of U2OS and MG-63 cell cycle by flow cytometry. Compared with the *miR-379* mimic NC group, the percentage of OS cells at the G_0_/G_1_-stage in the *miR-379* mimics group had a significant increase, while the percentage of OS cells at the S-stage significantly decreased (all *P*<0.05). Compared with the blank group, the percentage of OS cells at the G_0_/G_1_-, G_2_/M- and S-stages in the *miR-379* mimic NC, *miR-379* inhibitor NC, control shRNA and *miR-379* inhibitor + EIF4G2 shRNA groups were not statistically significant (all *P*>0.05). Compared with the *miR-379* inhibitor NC group, the percentage of OS cells at the G_0_/G_1_-phase in the *miR-379* inhibitors group had an obvious decrease, while the percentage of OS cells at the S-stage had an evident increase (all *P*<0.05). Compared with the control shRNA group, the percentage of OS cells at the G_0_/G_1_-phase increased, while the percentage of OS cells at the S-stage decreased in the EIF4G2 shRNA group (all *P*<0.05).

**Figure 6:** Cell cycles of U2OS and MG-63 cell lines detected by flow cytometry. (**A**) The cell cycle of U2OS cells in each group; (**B**) the cell cycle of MG-63 cells in each group; *n*=3; #, *P*<0.05 compared with the *miR-379* inhibitor NC group; *, *P*<0.05 compared with the *miR-379* mimic NC group; @, *P*<0.05 compared with the control shRNA group.

## Discussion

OS is the most common, primary malignancy with regard to bone [15]. Several studies have reported the significance of miRs in relation to OS including *miR-101, miR-26b* and *miR-30a* [16–18]. In the present study, it was established that *miR-379* exhibited a low level of expression in U2OS and MG-63 cell lines. In addition, inhibition in proliferation, migration and invasion of OS cells was observed when EIF4G2 was targetted.

Observations made during the present study indicated that *miR-379* was significantly down-regulated in OS cells and could inhibit the proliferation, migration and invasion of OS cells. In relation to previous reports and scientific literature concerning epithelial-to-mesenchymal transition (EMT), MiRs have been shown to regulate EMT and their effect on transcription factors and signaling pathways [11,19,20]. EMT is a process involving the transformation of epithelial cells into mesenchymal cells, featuring a loss of cell–cell adhesion and the acquisition of increased migratory and invasive capabilities [21]. EMT occurs in most tumorigenic cells, leading to increased invasion and metastasis in tumors [22,23]. Cancer cells usually undergo EMT before metastasis to distant organs and activate embryonic programs and pathways, which partially involve maintaining stem cell like characteristics [11]. Studies have noted the significant role of miRs in metastasis and cancer stem cell formation [9,24]. The expression of *miR-409-3p*, which belongs to the same cluster as *miR-379* does, is also down-regulated in OS. It is also associated with OS metastasis in suppressing OS cell migration and invasion [14]. *miR-379* can also regulate cyclin B1 expression and is decreased in breast cancer [25]. It has also been reported that *miR-379-5p* could inhibit migration as well as invasion in hepatocellular carcinoma cells by targetting FAK/AKT signaling pathways [10].

The most significant conclusion drawn from the present study was that *miR-379* could potentially act as a suppressor of OS. This could be showcased by directly targetting EIF4G2. Intriguingly, as our study revealed, the mRNA expression of EIF4G2 was significantly down-regulated in the *miR-379* mimics group and up-regulated in the *miR-379* inhibitors group. This highlighted the negative correlation in relation to the expression rate of *miR-379*. The dual luciferase reporter gene assay further confirmed that EIF4G2 was a target gene of *miR-379*. In addition, *miR-379* was found to significantly inhibit the proliferation, migration and invasion of OS cells. Translation of most mRNAs is regulated at the level of initiation, a process requiring the protein complex known as eukaryotic initiation factor 4F (EIF4F), which includes the cap-binding protein EIF4E, the scaffolding protein eukaryotic translation initiation factor 4 γ (EIF4G) and the ATP-dependent RNA helicase EIF4A [26,27]. The eukaryotic translation initiation factor 4, γ (EIF4G) is expressed in mammalian cells in two forms, namely, EIF4G1 and EIF4G2 [28,29]. Accumulating evidence has shown that disrupted translational machinery strongly contributes to cancer development and progression [27,30]. Translational deregulation occurs through modification of the expressions of proteins involved in translational initiation and/or changes in miR expression [31–33]. Recently, several studies have focussed on exploring the mechanisms underlying translational regulation via miRs [34,35]. Mazan-Mamczarz et al. [27] demonstrated that the down-regulation of EIF4G2 by siRNA decreased translation and cell proliferation and induced cellular senescence. Consequently, we hypothesized that the effect of miR-379 on OS progression may be due to its targetting EIF4G2.

One of the major limitations of the present study is the use of transient transfection of *miR-379* instead of stable expression in OS cell lines. Furthermore, knockdown *miR-379* in other non-cancerous osteoblastic cell lines should further substantiate its tumor-suppressing role in OS. To conclude, we established that the expression of *miR-379* was down-regulated in OS cell lines. In addition to this, the overexpression of *miR-379* was found to suppress OS cell proliferation, migration, invasion and tumour growth. The function of *miR-379* was mediated by the down-regulation of EIF4G2. The data collected and evaluated suggest that *miR-379* down-regulation may play various crucial roles in the development of OS. Thus, *miR-379* may serve as an effective therapeutic focus in inhibiting OS progression. Further studies are needed to investigate the clear roles that various miRs and their target genes play, in the development and progression of OS.

## Abbreviations

*C*_t_: cycle threshold
DLK1-DIO3: δ-like 1 homolog-deiodinase, iodothyronine 3
EIF4G: eukaryotic translation initiation factor 4 γ
EIF4G2: eukaryotic initiation factor 4GII
EMT: epithelial-to-mesenchymal transition
NC: negative control
OS: osteosarcoma
PI: propidium iodide
qRT-PCR: quantitative real-time PCR
